# Mobile Terminal Equipment and Methods of Martial Arts Movement Correction in Intelligent Physical Education Environment

This article has been retracted.

**DOI:** 10.1155/2022/7390836

**Published:** 2022-07-21

**Authors:** Meng Xu, Yaya Shi

**Affiliations:** ^1^Department of Physical Education, Honam University, Gwangju Metropolitan City 62397, Republic of Korea; ^2^Department of Physical Education, Gangneung-Wonju National University, Gangneung 25457, Gangwon-do, Republic of Korea

## Abstract

In recent years, the physical quality of middle school students in China has generally declined, which has attracted the attention of the state and the Ministry of education. With the development of Internet technology, China's physical education teaching environment has gradually become intelligent. This article mainly studies the mobile terminal equipment and methods of martial arts movement correction in the intelligent physical education environment. 21 young martial arts athletes were selected as the research objects. In the experiment, functional screening (FMS) was used to test the martial arts athletes, followed by FMS tests and scores. A video camera was used to record the motion test from the subjects' sagittal and frontal planes. Using wireless sensor technology to collect the athletes' motion signals, after the twelfth week, the FMS, SEBT, and the number of successful routines were tested on the two groups of athletes, respectively. The pre-test data and the post-correction data of the two test indicators were compared and analyzed. There is no significant difference. The necessary statistics and integration of the obtained data are carried out by using the calculation methods in sports statistics. The experimental data showed that the average total scores of FMS screening test of Changquan athletes and Taijiquan athletes were 14.71 ± 1.52 and 16.20 ± 1.32, respectively. The results of the research on the mobile terminal equipment and methods of martial arts movement correction in the intelligent sports environment show that the mobile terminal equipment can improve the independent training ability of athletes, and at the same time has a good correction effect on irregular movements.

## 1. Introduction

With the rapid development of China's physical education and the deepening of the reform of school physical education curriculum, including theoretical courses and technical courses, the requirements of schools for physical education teachers are also increasing. Network technology has not only changed our daily life, but also changed our physical education teaching mode. Now, the teachers and students who are teaching college physical education are feeling the change of teaching mode brought by network technology. For most students, asymmetric movements and bad movement patterns tend to aggravate the formation of their bad body posture, resulting in sports injury, thus affecting the normal growth and development. Therefore, it is urgent to correct the bad movement patterns of college students. The smart sensor can automatically collect data and preprocess the data.

In competitive sports, coaches, as the backbone of guiding sports activities, shoulder the important mission of leading and guiding athletes to complete sports competitions. Therefore, coaches are required to correctly grasp the laws of sports activities and deal with the relationship between competition and sports training. The occurrence of sports injury is mostly due to the long-term failure to correct the compensatory movement mode of athletes in daily training and competition, resulting in functional changes of a certain joint, which will affect other normal physical functions in the long run. Through the intelligent sensor it can quickly and efficiently capture the athletes' nonstandard movement signal, and then transmit the signal to the mobile terminal device, so as to improve the quality of athletes' action and reduce the occurrence of sports injury. The development of network technology has changed the traditional physical education model, making physical education more intuitive and efficient; the means of education have been updated, and the rich sports information resources on the Internet and the convenient and fast information acquisition methods have provided the reform of physical education methods in an excellent condition.

In the stage of motion correction, the primary problem is how to immediately judge whether the motion is standard or not, and correct the irregular motion. DAMACENA tested a theoretical model. He conducted a survey of 328 judo players in the Brazilian stadium. He analyzed the data using PLSmart software, which uses the partial least squares method. He found that market demand positively affects the perceived benefits and value, as well as the satisfaction and commitment of judo members. He also found that perceived benefits have a positive impact on perceived value, which positively triggers satisfaction, thereby increasing the practitioner's commitment. Although his research has certain reference value, it is not accurate enough [1].

Mayorga Vega mainly studies the influence of the development and maintenance plan based on physical education on the objective and perceived health-related physical health of high school students. He randomly divided a sample of 111 to 12–14-year-old students from six classes into an experimental group (*n* = 54) or a control group (*n* = 57). At the beginning and end, he measured the students' objective cardiopulmonary fitness (20 meter shuttle test), objective muscle fitness (leg flexion and extension test), and perceived physical fitness (International adaptability scale and contour map assessment scale), respectively. Although his research is accurate, it is not comprehensive [2].

Pesce C's research aims to verify whether the life skill plan (PE) in sports has a positive impact on physical health, motor skills, and executive cognitive functions, and whether the final physical and sports results are introduced by the improvement of life skills and executive functions guide. Although his research can make a reasonable evaluation of experimental subjects, it lacks experimental data [3].

Tirunagari S believes that due to the rapid change of contrast agent in the DCE-MR image sequence, the commonly used intensity-based image registration technology is likely to fail. He proposed a novel, automatic motion correction method without registration based on a reconstruction variant of window mode and dynamic mode decomposition (WR-DMD). The method he proposed was validated on the kidney DCE-MRI dataset of ten different healthy volunteers. He uses image sequences generated by WR-DMD for block matching block evaluation. Although his research can avoid artificial interference, it is not accurate [4].

Through the introduction of smart phones and other mobile terminals into the teaching of college physical education, it can increase students' interest in learning, improve students' learning efficiency, optimize students' management, improve the teaching quality of college sports major, reduce the teaching burden of teachers, and improve teaching efficiency. At the same time, it can better complete the teaching task while reducing the students' learning pressure and teachers' teaching burden. At the same time, with the help of the Internet of things and wireless sensors, students' irregular martial arts movements can be corrected in time to improve the teaching level of teachers and the learning quality of students. The rapid development of network communication industry has created favorable conditions for the teaching of physical education in colleges and universities with mobile terminals, which makes the teaching work of physical education more convenient and flexible. The innovation of this paper lies in the combination of sports and martial arts with mobile terminal equipment, which has certain innovation and practicability [5].

## 2. Martial Arts Movement Correction Mobile Terminal Equipment

### 2.1. Internet of Things

The Internet of Things is a derivative product of the Internet. It is also called a sensor network. It is based on the Internet. It allows any item to be connected and connected in the Internet, and realizes the relationship between things and the Internet under the requirements of limited agreements. The mutual information exchange and communication, and finally achieve modern functions such as positioning, detection, tracking and management of items, including intelligent identification. In addition, RFID electronic tags also support the exchange and communication of information about items in the Internet of Things anytime and anywhere, with rich and powerful functions [6, 7].

The architecture diagram of the Internet of Things is shown in Figure 1. From a technical perspective, the modern Internet of Things is divided into three main levels at the overall design structure level: perception layer, transmission layer, and business layer. Among them, the most important perception layer mainly revolves around RFID electronic tags and RFID readers, which can perceive and obtain real-time information of enterprise goods. Then, through the transmission layer network sense, the cargo information obtained by the perception layer is implemented and transmitted, which provides an information basis for the construction tasks of the business layer, and at the same time implements effective data processing, and finally achieves the practical purpose of controlling the cargo. If each node has its own data communication capabilities, it can receive and forward data, and send or forward data directly between nodes, without relying on base station facilities, then this problem will be solved to a certain extent. The network that can be used as relay routing is called ad hoc network [8].

The topology of the Internet of Things describes the wireless communication relationship between various nodes in the network, and is the basis for the design of various network communication protocols and routing protocols. Designing a high-quality, robust, and efficient topology is of great significance to the substantial improvement of the network's transmission delay, life cycle, and throughput. In scale-free topology, the degrees of all nodes conform to the power-law distribution. Therefore, the most important way to verify the scale-free characteristics of the topology is to analyze and prove the degree distribution in the topology. In order to approximate the degree distribution of nodes in BA topology, we assume that time is not discrete points but continuous. Similarly, it is assumed that the degree of the node may not be an integer, but continuously change [9, 10]. The degree of a node is a branch of a node. If there is one branch, the degree of a node is 1. By analogy, a node is a term that refers to a type of device, which can be a host, a server, or a switch or router that constitutes a transmission network, firewall, etc [11]. The conversion rate of node degree is

(1) $$\begin{array}{c} m\prod_{i}=\frac{md_{i}\left(t\right)}{\sum_{j=1}^{m_{0}+t}d_{i}\left(t\right)}=\frac{md_{i}\left(t\right)}{2mt}=\frac{d_{i}\left(t\right)}{2t}. \end{array}$$

In the formula, *d*_*i*_(*t*) is the degree of node *i* at time *t*.

For the time continuous analog signal *x*(*t*) and the frequency spectrum relationship *X*(*f*) can be expressed as:

(2) $$\begin{array}{c} x\left(t\right)=\int_{-\infty }^{+\infty }X\left(f\right)e^{i2\pi ft}\text{d}f,\\ X\left(f\right)=\int_{-\infty }^{+\infty }x\left(t\right)e^{-i2\pi ft}\text{d}f. \end{array}$$

*x*(*nTs*) can completely determine *X*(*f*) to determine *x*(*t*), and its expression is as follows:

(3) $$\begin{array}{c} x\left(t\right)=T_{s}\sum_{n=-\infty }^{+\infty }x\left(nT_{s}\right)\int_{-1/2T_{s}}^{1/2T_{s}}e^{i2\pi f\left(1-nT_{s}\right)}\text{d}f. \end{array}$$

### 2.2. Martial Arts Movement Correction

The human body is a complex interaction of the whole, bad posture is not only the appearance of beauty, but also a deep sense of physical health problems. If we do not pay attention to the bad body posture, it is easy to affect the physical health of the whole person, and then cause serious trouble to their normal life. Children and adolescents are in the peak period of growth and development; good body posture can provide a stable support and protection environment for the normal growth and development of their tissues and organs. From the perspective of biomechanics, it is found that the force of human body is very similar to that of buildings. When the straight line of the center of gravity of human body is vertical to the ground, the influence of gravity on the muscles and joints of human body is the least. In this position, the gravity is evenly distributed on the bones, joints, muscles, and ligaments of the human body, so each muscle needs only the minimum force for contraction or relaxation, and each ligament is in a moderate stretching state. The whole human body is in a perfect balance point. On this basis, the efficiency of human body movement is the highest, and the risk factor is the lowest. The stability of this balance can only be achieved by the coordinated effort of muscles in all parts of the human body [12, 13].

Participating in training will have the risk of sports injury, and the premise of sports injury is that there are problems in the movement mode in the process of sports, which requires correcting the action mode to avoid the occurrence of injury. The ultimate goal of corrective training is to enable people with limited physical activity to recover the basic activity ability of all parts of the body, and be able to control the movements of all parts of the body freely. The most basic use of functional training is to prepare athletes for their sport. Functional training employs concepts articulated by specialized coaches to train speed, strength, and explosiveness to improve athletic performance and reduce injury. The purpose of functional training is to restore the most essential function of the human body. Its FMS test also serves for functional training, helping assessors to formulate training correction plan according to the problems existing in the subjects' exercise mode, and guide functional training [14, 15]. Functional training is based on the functional structure of human body and the basic theory of sports anatomy, sports physiology, and neurology. It guides the neuromuscular skeletal system to combine the power chain system in the frontal, sagittal, and horizontal planes of the human body, so as to improve the body's motor function as a whole. Functional training emphasizes multi joint, multi-directional, and integration of proprioception, and aims at the high efficiency of movement mode and the economy of energy use in the process of sports [16, 17].

Correction training follows the pyramid principle from bottom to top, that is: joint flexibility and stability, muscle strength and symmetry, special technical training, so that the key points of each project training are different. The first link is the improvement of flexibility. Only by opening the joint flexibility can we have a larger range of motion and space, so that the range of action can be increased, and the participants can be free from the constraints of joints when completing specific actions. The second link is stability. Only with strong core and overall stability can we control the body well when completing specific actions, the last is symmetrical exercise. Only by paying attention to the symmetry of muscle force in the process of training and ensuring the participation and coordination of left and right muscles at the same time, can we effectively avoid the phenomenon of muscle compensation and imbalance of strength development. Only when the movement mode is optimized can the sports ability be improved [18, 19].

### 2.3. Mobile Terminal Equipment

First, a suitable chaos is selected and the image is encrypted by the generated chaos sequence. Then, an initial key with plaintext features can be generated from the plaintext image information, using the chaotic system as an intermediate key generator. After quantization, sequence data and image data can be reversibly operated. Finally, the randomness of the chaotic system diffuses to the entire plaintext image to generate an encrypted image [20]. Usually the operation is through XOR operator or addition operator and so on. The decryption operation is also very simple. As long as the same chaotic sequence is generated by the same method, the original plaintext image can be obtained by the reverse operation again. The number of initial values and initial parameters of chaotic system often determines the key space of encryption system. Therefore, in the process of key generation, more parameters and more complex chaotic system are often needed as key generator to improve the security of the algorithm [21, 22].

The far-field formula of rectangular microstrip antenna and the pattern functions of E-plane and H-plane are as follows.

(4) $$\begin{array}{c} F=\frac{\varepsilon_{0}}{4\pi }\left[\iint_{S_{1}}M_{S_{1}}\left(r^{\prime }\right)\frac{e^{-j\beta R_{1}}}{R_{1}}ds^{\prime }+\iint_{S_{2}}M_{S_{2}}\left(r^{\prime }\right)\frac{e^{-j\beta R_{2}}}{R_{2}}ds^{\prime }\right]. \end{array}$$

In the formula, *S*_1_ and *S*_2_ represent the caliber surfaces of the two slits, and *R*_1_ and *R*_2_ represent the distance from the small surface element on the two caliber surfaces to a point in the far space. In order to reduce the number of microstrip antennas and reduce the complexity of antenna design, the navigation antenna of mobile terminal usually works in dual band or multi band. Nowadays, stacked radiation patch structure is widely used in antenna design: two resonators are generated by superposition of two layers of radiation patches to make the antenna work at the resonant frequency corresponding to the two resonators. This method can make the design of multi band and broadband antenna easier. At the same time, using this method will inevitably lead to the introduction of multi-layer dielectric layer or different types of dielectric layer into the dielectric substrate of the antenna, which will increase the height of the antenna and increase the difficulty of manufacturing. In addition, slot antenna is also very popular in antenna design, because the antenna designed with this structure is easy to achieve a wide impedance bandwidth [23].

## 3. Martial Arts Movement Correction Experiment

### 3.1. Subjects

Select 21 young martial arts athletes as the research objects. The basic information of the subjects is shown in Table 1. Among them, 14 are male athletes and 7 are female athletes. The subjects' special training time ranges from 4 to 15 years; the sports level is national level one or two; the average age is 19.24 ± 1.221; the athletes are in good health, and there is no major torso injury or surgery in the past 6 months The limitation of athletic ability does not rule out a history of past injuries [24, 25].

### 3.2. Test Method

Functional screening (FMS) was used to test Wushu athletes, and then FMS was tested and scored. The intragroup correlation coefficient (ICC) statistical method was used to evaluate the reliability of on-site scoring and video scoring for FMS. The results showed that the reliability of field scoring and video scoring was highly consistent (ICC = 0.92, 95% CI = 0.855) and repeatability. Before the test, it is necessary to explain and train the personnel of the test group to make them fully understand and master the test process. The test was conducted at the same time. First, the subjects were explained to make them understand the test content correctly. Then, the warm-up activities were carried out first, and then the test results were recorded. Finally, the test data were sorted out. After the test, the data was sorted out [26].

Before the experiment, FMS, SEBT test, and routine exercise success rate test of Changquan group and Tai Chi group were carried out, and the initial test data of the two groups before correction were recorded. Then, independent sample *t*-test was conducted between Changquan group and Tai Chi group, and the functional rules between the two items were analyzed, and the vertical intragroup comparison was conducted, the symmetry of limb function was analyzed. After the beginning of the experiment, correction training was carried out three times a week. After the 12th week, the two groups of athletes were tested for FMS, SEBT, and the number of successful routines. The differences between the pre-test data and the corrected data of the two groups were compared and analyzed [27].

### 3.3. Signal Collection and Motion Correction

1. During the test, wireless sensor technology was used to collect the motion signals of the athletes, and the camera was used to record the entire training process of the research subjects.
2. After the training, research the training videos of all subjects. Upload the athlete's irregular action clips to the mobile terminal device. The structural frame of the equipment is shown as in Figure 2. Athletes can reserve training time on the terminal, and the training content can be clearly played on the display of the device. During training, the pressure sensors on the arms, legs, and feet continuously collect pressure signals, and upload the collected data to the controller to analyze the trainee's posture based on the pressure data. When the trainee's posture is wrong, the system automatically sends out the warning sound reminds the trainee to adjust the posture. When the pressure detected by the corresponding pressure sensor returns to a reasonable value, the warning sound stops to achieve the purpose of continuing to maintain the correct action; when the training time is up, the voice alarm will send an alarm signal. It prompts the end of the training, and at the same time replays the recorded training video on the touch screen, analyzes the training actions, and prompts the trainees to correct errors and irregular actions [28, 29].

### 3.4. Data Processing

The necessary statistics and integration of the obtained data are carried out by using the calculation methods in sports statistics. All the test index data before and after the experiment were input into the computer, and then imported into the spss22.0 statistical software via Excel for analysis. The analysis results were described by the mean ± standard deviation (*M* ± SD). The independent sample *T* test was used to analyze the FMS scores of martial arts students of different genders. *P* < 0.05 or *P* < 0.01 are both statistically significant [30].

## 4. Martial Arts Movement Correction Analysis

### 4.1. Analysis of Test Results

The purpose of FMS test is not simply to know whether the subjects can achieve 21 points or complete 3 points, but to focus on the individuals with 0 points, 1 items, asymmetry, and the total score of FMS less than or equal to 14 points. A single score of 0 indicates that the subject has pain in a certain part of the body, and a single score of 1 indicates that the subject's body is asymmetric or severely limited in functional movements. Corrective training emphasizes training action rather than muscle training. It stimulates and perfects the use and feedback of the central nervous system to muscles through reasonable training methods. It emphasizes the participation of proprioceptive receptors in the completion of specific actions, so that the nerves can actively mobilize various tissues and muscles of the body to complete the action in a correct way. Its essential function is to improve the imbalance, asymmetry, and uncoordinated development of the body through the correction of technical movements, and restore the body's original role. Therefore, the participation of each muscle group is emphasized in the training, including: core muscle group, active muscle group and auxiliary muscle group, large muscle group and small muscle group, surface muscle group and deep muscle group, participating in the formation of movement harmoniously. It is absolutely not allowed to appear the phenomenon that a single muscle or muscle group exerts force alone, which leads to the imbalance of body compensation and muscle development.

Table 2 shows the data comparison between the FMS test indicators of the Changquan group and the Tai Chi group. From the data in the table, the average total scores of the FMS screening test for Changquan and Tai Chi athletes are 14.71 ± 1.52, 16.20 ± 1.32, respectively. It is not difficult to see from the data that the Tai Chi group is significantly higher than the Changquan group, *P* < 0.01, there is a very significant difference between the two groups, in the squat test, *P* < 0.05, indicating that there is a significant difference between the two groups, the Tai Chi group scores significantly higher than the Changquan group; the shoulder joint is flexible in the sex test, *P* < 0.01, indicating that there is a very significant difference between the two, the Tai Chi group scores significantly higher than the Changquan group; in the hurdle step, front and rear legs squatting, trunk stability push-up, and torsion stability action test. In the middle, *P* > 0.05, indicating that there is no significant difference between the Changquan group and the Tai Chi group; the analysis of the data shows that all the tested athletes have lower scores in the trunk stability push and torsional stability test. In this study, the average score of the total scores of the two groups of athletes in the FMS test was above 14 points, indicating that the probability of sports injuries in the two groups of athletes during training is not very large, and the overall condition of the Tai Chi group athletes is better in avoiding sports injuries. In the Changquan group, this may be related to the action characteristics of the two types of boxing. The movements in the Changquan routines are mostly fast and coherent, the posture stretches quickly and powerfully, the movement is fast and quiet, the rhythm is clear, the ups and downs are more flexible, and the long-strike speed is active. The Tai Chi movements are mostly slow and soft. The lightness is continuous, and most of the exercise is in a half-squatting state, with strong leg strength.

The movement changes of the experimental subjects before and after corrective training are shown in Table 3 and Figure 3. It can be seen that before the corrective training, the athletes' test scores were generally low, with the highest score of 17.7; after the corrective training, the athletes' movements were generally standardized, and the test scores were greatly improved, with the highest score of 20.0.

As can be seen from Figure 3, through the correction training, the movement changes after correction are generally improved, and the improvement range is large. The movement changes of athletes before correction are always between 9.8 and 17.7, and the changes of athletes after correction are 8.8. −20.7, indicating that the corrective effect is obviously effective [31].

### 4.2. Analysis of Motion Correction Mode

The results of action mode screening are shown in Figure 4. Judging from the overall screening of athletes' action patterns, in the three screening results of squats, trunk stability push-ups, and rotation stability, it is found that athletes have a larger proportion of 3 points, 75%, 62.5%, and 75%; while the proportion of athletes who scored 3 points in the screening of hurdles, squats, shoulder flexibility, and supine straight legs and knee lifts is relatively small, 37.5%, 25%, 12.5%, and 25%, respectively. In addition, the proportion of athletes who scored 0 in the screening of shoulder joint flexibility and trunk stability is relatively small, both 12.5%; there is no occurrence in the screening of squats, hurdles, squats, and rotation stability. If an action pattern similar to the hurdle-crossing and stepping action is bad, the body's limbs movement function will appear asymmetry, resulting in sports injuries. The scores of the college students' hurdle-crossing and stepping action test before and after the two classes are matched. After the sample *T* test, it was found that there were extremely significant differences between the two classes before and after the experiment, indicating that fitness yoga can improve the bilateral flexibility and stability of the hips, knees and ankles, and enhance the stability of the pelvis and the core of the body. And control ability, improve the scores of college students' hurdle-crossing action test, and correct bad hurdle-crossing action. Therefore, from the perspective of the quality of movement completion, the completion of the four movement modes of hurdle step, straight lunge squat, shoulder flexibility, and active straight knee lift is better than that of trunk rotation stability movement mode. From the point of view of the scores of the opposite limbs of the five action modes, the score of the dominant side limb is lower than that of the nondominant side, indicating that the muscles of the dominant side limb are more tense than the nondominant side, which makes the dominant side limb joints flexible to a certain extent. Sex is limited, and the stability is affected accordingly.

### 4.3. Role of Mobile Intelligent Terminals in the Learning of Sports and Martial Arts in Colleges and Universities

The application of mobile smart terminals before class is mainly focused on publishing class notifications and publishing preview content. Due to the portability and popularity of smart phones, students will receive all kinds of information as soon as the teachers release it. Also because of the portability of smart phones, students can preview what they will learn anytime, anywhere. Digital teaching materials can be used during class, making it easier for teachers to give lectures. Students can also inquire about teaching materials through smartphones to make the learning process more active. In the course of class, students can take class notes by shooting, recording, and taking photos with their mobile phones. In the practical course, you can also use the smart phone's camera, photo, and other functions to help students learn sports. For example, when a student completes an action, he uses his mobile phone to take a picture of the action. The student repeatedly observes the action he has completed to discover and correct his own mistakes. At the same time, for some difficult movements, the physical education teacher can only do the movements over and over again, and cannot explain the movements separately. Then using the dynamic display, the difficult movements can be broken down step by step and the true face of the movement can be restored. It is difficult for teachers to demonstrate and explain the movements. With the help of dynamic demonstration, the movements can be completely reproduced. Students can master difficult movements accurately, and it is not difficult to learn difficult movements.

The total FMS scores of the subjects before and after the correction intervention are shown in Figure 5. It can be seen that the percentages of people with total scores in the 10–15 score segment are significantly reduced, and the percentages of people who score are mainly concentrated in the 16–18 score segment. The number of scores with 17 points and 18 points has increased significantly. It shows that the total score of FMS has been significantly improved after intervention training. The action design for comprehensive correction of scoliosis, by changing the external force environment of the patient, achieves the relative stability of the internal structure, improves the core stability, and finally achieves a balanced state of reshaping the spine with uniform force.

### 4.4. Effect of Corrective Training on Body Shape

Before the experiment, during the experiment, and after the experiment, the subjects were tested for the physical fitness of the body shape, quality, and skills. The test results are shown in Figure 6. When there was no significant difference in the indicators (*P* > 0.05), the longer the time, the better the performance in body shape. There are a lot of training methods and means that can be improved in the correction training of young football players. We should further improve and pay attention to the training of physical fitness in the youth stage. Especially in the youth football correction training methods, we should not ignore the sensitive period and other important factors in the process of physical training. Only by arranging the tasks, contents, means, methods, and loads of physical training according to the nature of the development stage of sports, can we achieve the maximum development in some factors and ensure the best state of the body when entering the stable period. The training means and methods improve the quality of young football players in order to improve their training level.

During training and competition, athletes need to keep changing speeds and changing directions to gain initiative and increase scoring opportunities. This test action attempts to place the body in a special exercise posture to screen out the functional problems of various parts of the body when the action is completed. It specifically examines the body's load in the hip posture; in the mobile state, the body's stability and dynamic postural stability. The results showed that the athletes performed relatively stable in the action evaluation, and the number of people who scored 1 point was relatively small; most athletes showed significant forward movement of the torso center of gravity, slight body swing, crossbar not close to the body, and ankle joint shaking when squatting.

## 5. Conclusions

This paper mainly focuses on the mobile terminal equipment and methods of martial arts movement correction under the intelligent sports teaching environment. The weakness of body quality, flexibility, and muscle of male and female students are mainly manifested in weakness of body quality and flexibility of shoulder. Among the weak qualities checked out, trunk stability push-up and trunk rotation stability had the lowest scores, with an average of about 1.5 points, indicating that it is particularly important to strengthen and improve students' core muscle strength and body coordination.

Mobile terminal equipment can improve students' autonomous learning ability. Students learn sports through their own mobile devices, with great autonomy and flexibility. As long as there is a network place, you can learn anytime and anywhere. Students can use fragmented time to learn physical education courses, improve their independent learning ability, exercise their ability of autonomous learning, and enhance their initiative in learning sports.

Regarding the action sequence can be regarded as a collection of bone data, comparing the difference between the two action sequences is regarded as comparing the difference in the characteristics of the action sequence; the direction of the limbs formed by the adjacent joints is used to correct the action. Then, based on the use of dynamic time warping method to align the action time series, the action similarity is judged based on the feature vector and the cosine similarity. Finally, with the help of the angle feature to express the movement trajectory, the overall movement comparison analysis result is obtained. The application of artificial intelligence technology has been integrated into all corners of human life, including learning, teaching, and decision-making tools, and then to management systems or platforms, so as to give full play to its corresponding functions, which also brings new opportunities for the development of smart sports. Because the data in this paper is not enough, the experimental research is too one-sided, and it will be continuously improved in the future study.

## Figures and Tables

**Figure 1:** Architecture diagram of the internet of things.

**Figure 2:** Frame structure of mobile terminal equipment.

**Figure 3:** Movement changes before and after correction training.

**Figure 4:** Action mode screening results.

**Figure 5:** The total scores of subjects before and after correction intervention.

**Figure 6:** Test results.

**Table 1:** Basic information of subjects.

Gender	Age	Height	Body weight	BMI	Training time
Male	18.69 ± 2.36	171.22 ± 12.41	72.15 ± 6.79	23.10 ± 2.76	6.6 ± 8.4
Female	19.21 ± 1.08	165.29 ± 7.49	74.21 ± 7.16	19.81 ± 1.83	5.1 ± 9.9

**Table 2:** Comparison of data between two groups of FMS test indicators.

Test index	Changquan group	Tai chi group	*t*	*P*
Squat	2.17 ± 0.57	2.70 ± 0.48	−2.610	0.014
Hurdle step	2.08 ± 0.28	2.10 ± 0.32	−0.152	0.881
Squat	1.92 ± 0.58	1.90 ± 0.74	0.070	0.944
Shoulder flexibility	2.50 ± 0.51	2.90 ± 0.32	−2.769	0.010
Trunk stability push	1.17 ± 1.01	1.60 ± 0.84	−1.287	0.213
Torsional stability	1.88 ± 0.45	1.90 ± 0.32	−0.160	0.874

**Table 3:** Movement changes before and after correction training.

1	2	3	4	5	6	7	8	9	10	11	12	13	14	15	16	17	18	19	20	21
10.5	10.7	14.7	9.8	13.7	12.7	15.4	11.1	12.6	11.7	17.7	17.7	9.9	14.5	12.1	17.3	12.5	10.6	14.1	11.4	13.6
17.4	19.2	10.5	17.0	16.2	20.0	10.2	20.7	13.7	10.1	11.2	9.6	14.5	17.2	10.8	10.4	12.0	17.8	11.6	18.5	8.8

## Data Availability

No data were used to support this study.
